# Epileptic Seizure Detection Using a Hybrid 1D CNN-Machine Learning Approach from EEG Data

**DOI:** 10.1155/2022/9579422

**Published:** 2022-11-29

**Authors:** Fatima Hassan, Syed Fawad Hussain, Saeed Mian Qaisar

**Affiliations:** ^1^Faculty of Computer Science and Engineering, G. I. K. Institute, Topi, Pakistan; ^2^School of Computer Science, University of Birmingham, Birmingham, UK; ^3^Electrical and Computer Engineering Department, Effat University, Jeddah 22332, Saudi Arabia; ^4^Communication and Signal Processing Lab, Energy and Technology Research Center, Effat University, Jeddah 22332, Saudi Arabia

## Abstract

Electroencephalography (EEG) is a widely used technique for the detection of epileptic seizures. It can be recorded in a noninvasive manner to present the electrical activity of the brain. The visual inspection of nonlinear and highly complex EEG signals is both costly and time-consuming. Therefore, an effective automatic detection system is needed to assist in the long-term evaluation and treatment of patients. Traditional approaches based on machine learning require feature extraction, while deep learning approaches are time-consuming and require more layers for effective feature learning and processing of complex EEG waveforms. Deep learning-based approaches also have weak generalization ability. This paper proposes a solution based on the combination of convolution neural networks (CNN) and machine learning classifiers. It preprocesses the EEG signal using the Butterworth filter and performs feature extraction using CNN. From the extracted set of features, the approach selects only the relevant features using mutual information-based estimators to reduce the curse of dimensionality and improve classification accuracy. The selected features are then passed as input to different machine learning classifiers. The suggested solution is evaluated on the University of Bonn dataset and CHB-MIT datasets. Our model effectively predicts 2, 3, 4, and 5 classes with accuracy of 100%, 99%, 94.6%, and 94%, respectively, for the Bonn dataset and 98% for CHB-MIT datasets.

## 1. Introduction

Epilepsy is a prevalent chronic neural disorder caused by irregular electrical discharges, which are known as seizures. These seizures can result in abnormal activity of the brain, unconsciousness, recurrent convulsions, serious injuries, and in some cases even death. About 50 million people worldwide are diagnosed with epilepsy with the biggest impact on children and adults aged 65–70 years [1]. Eighty percent of epileptic seizures can be controlled if they are correctly and timely diagnosed [2]. Electroencephalography (EEG) is a widely used technique for epileptic seizure detection. The visual analysis of these highly complex EEG signals is a hectic and time-consuming procedure [3]. It can also lead to diagnostic errors due to fatigue or the physician's lack of concentration. In addition to recording brain activity, the EEG signals include a significant amount of random noise which can affect the performance of the model [4]. Therefore, it is important to have an effective, accurate, and timely diagnosis of epileptic seizures in order to initiate medication and antiepileptic drug therapy to minimize the risk of potential seizures [3, 5]. These challenges inspired many researchers to find an effective and automated solution for the real-time detection of epileptic seizures.

Given the EEG waveforms, feature extraction and classifier training are the two fundamental processes for automatic seizure detection. Researchers have experimented with different combinations of signal preprocessing, feature extraction, and feature selection methods coupled with different classification algorithms. For instance, in [6], Martis et al. used empirical mode decomposition (EMD) to obtain eight intrinsic mode function (IMF). From these IMF's, 32 features were extracted and ranked using analysis of variance (ANOVA). They were able to classify normal, interictal, and ictal classes with 93.55% accuracy using a classification and regression tree (CART). Another study in [7] used recurrence quantification analysis (RQA) as a feature extraction algorithm in combination with an SVM classifier. Ein Shoka et al. [8] extracted statistical features. They selected three channels from the multichannel CHB-MIT database based on the variance.

Wavelet transforms have been considered efficient feature extractors and are therefore a widely used feature extractor for interpretation of transient signals. The work in [9] has used cross-information potential (CIP) methods along with tunable-Q wavelet transform (TQWT) for mining features which are then fed to random forest (RF) classifier. Alickovic et al. [10] used multiscale principle component analysis (MPCA) for signal denoising. For feature extraction, wavelet packet decomposition (WPD) has been used. Others, such as in [1], used Chebyshev IIR filter for noise removal and discrete wavelet transform (DWT), which decomposes the filtered signals into five sub-bands. They have used only delta sub-band for feature extraction and applied thresholding to determine the noisy part of the signal. In the final stage of classification, they have used an artificial neural network (ANN) and a support vector machine (SVM) [11] and also used DWT to extract temporal and spectral features, which were then sent to temporal and fuzzy classifiers.

ML-based classification models require large a number of samples for feature extraction. Manual extraction of these features requires domain knowledge and often results in the loss of some important details. Deep learning-based techniques, especially CNN, have been widely used for epilepsy classification. They overcome the limitations of ML-based methods and do not require feature extraction and selection. They have the ability that they can automatically perform feature extraction by learning the internal representation of the data, but these deeper networks can be difficult to converge. Like in [4], Acharya et al. trained a 13-layered deep CNN for a 3-class problem i.e., normal, interictal, and ictal. They obtained accuracy, specificity, and sensitivity of 88.7%, 90%, and 95% on the University of Bonn Dataset. Ullah et al. [12] proposed an ensemble-based technique that consists of one-dimensional pyramidal CNN models and predict the class label based on consensus. Data augmentation schemes have been used to overcome the limitations of small dataset. The performance of the proposed architecture is evaluated on University of Bonn datasets. In [13], authors proposed a new feature fusion CNN model for the classification of normal, preictal, and seizure states. This model is based on a dilated convolution kernel and is an improved version of conventional CNN. Their main focus was on reducing the parameters. This model is also tested on three classes of the Bonn University dataset. Another study in [14] used all five classes of the Bonn dataset. They obtained two-dimensional frequency-time scalograms from raw EEG signals using continuous wavelet transform (CWT) and then trained CNN on these scalograms. A study conducted in [3] proposed a novel one-dimensional deep neural network consisting of a series of convolutional layers, a batch normalization layer, a dropout layer, and a max-pooling layer for robust detection of epileptic seizures. The authors in [15] also worked on a 3-class problem. They implemented a hybrid model of CNN and the long short-term memory (LSTM) network. In [16], Srinath et al. used EMD to decompose signal into six IMFs. The intrinsic features were computed from these sub-bands. These features along with IMF sub-bands were fed to CNN for classification in order to achieve higher classification accuracy. This method is tested on the 2-class problem of the CHB-MIT dataset.

Another study conducted in [17] decomposed the EEG signals into frequency bands using Fast Fourier Transform (FFT). The spectral power and mean spectrum amplitude are computed for all bands and fed to the LSTM for binary classification. Hu et al. [18] used local mean decomposition to extract features and then passed them to Bi-LSTM for classification. A research study in [19] presented a network that employs contrastive supervised learning and replaces the multiplication with the addition operation in traditional convolutional networks. The presented model was tested on the CHB-MIT dataset and obtained an AUC (area under the curve) score of 94.2%. This score represents the capability of the model to distinguish between the classes accurately.

From the literature, it is observed that deep learning-based models consisting of approximately 10 or sometimes even more than that number of layers is required for accurate classification. For multiclass problem, deeper architectures are designed using multiple dense layers, which results in thousands of parameters. The research study in [4] used 13-layers for classifying three classes of epileptic seizures. Such models are computationally and spatially expensive. On the other hand, machine learning-based models are easier to learn and give competitive accuracies with the right features. However, the feature extraction and selection require domain knowledge and may need to be tuned for different datasets. An appropriate selection of features for model training is one of the most crucial steps. Deep learning models can do this step automatically.

### 1.1. Main Contribution

In the literature, most of the related studies have reported variable classification results for different noninvasive EEG epileptic seizure datasets. The DWT was found to be an effective decomposition approach for the seizures detection. However, different researchers employed a variety of algorithms to extract features from the approximate and detailed coefficients, obtained through the DWT. There is no general feature extraction algorithm presented that can work for a variety of EEG datasets. These limitations in the literature motivated us to propose a method that can work for multiclass, multisubjects, and multichannel EEG datasets.

The main contributions of this paper are as follows:

- This paper proposes a model which uses the automatic feature extraction capability of neural networks and machine learning algorithms for the prediction of seizures.
- An effective method is suggested for classification of multiclass, multisubjects, and multichannel EEG signals by using the Butterworth filter, DWT, and CNN for noise removal and feature extraction. Approximate and detailed coefficients are extracted from Butterworth filtered EEG signals using Daubechies order 4 discrete wavelets transform to remove the redundant information. The hand crafted extraction of features from sub-bands in replaced by the automatic feature extraction capability of CNN.
- From these extracted features, the features which have high information gain are selected using the mutual information. The selected features are fed to different machine learning classifiers for training and accuracy was reported on two, three, four, and five classes.

The model works by (i) Acquiring EEG signals from human brain which are preprocessed using Butterworth filter to filter out noise. (ii) These preprocessed and filtered EEG signals are decomposed into 5 sub-bands using Daubechies order 4 discrete wavelet transform. (iii) The result is then fed to the convolutional network layer for feature extraction. (iv) Mutual information (MI) estimator is used for selecting the most relevant features among these learned features of CNN, and (v) The result is then passed to different machine learning classifiers. The performance of proposed model is evaluated on the Bonn Dataset and CHB-MIT dataset. It permits to evaluate the suggested method performance for the case of for multiclass, multisubjects, and multichannel EEG datasets. Multiple evaluation metrics are used for model evaluation such as precision, recall, and *F*1-score.

## 2. Materials and Methods

The block diagram in Figure 1 describes the approach followed in this paper. The model's performance is then evaluated on two, three, four, and five classes.

In the above figures, A and D represent the approximate and detailed coefficients. DWT decomposes the preprocessed signals into approximate and detailed coefficients from which features are extracted.

### 2.1. Dataset Description

#### 2.1.1. University of Bonn Dataset

The dataset used in this research is of EEG segments obtained from Bonn University, Germany [20]. These signals are recorded from a 128-channel amplifier system in a noninvasive manner and using 12-bit analog to digital converter. Each set has a total of 100 single-channel EEG signals with 4097 sample points per channel. Every signal has duration of 23.6 seconds and a sampling frequency of 173.61 Hz. The dataset consists of five sets of EEG signals: Z, O, N, F, and S which are denoted as A, B, C, D, and E in this paper. The recordings in ‘A' and ‘B' sets are obtained from heathy patients with eyes open and closed whereas the remaining three records contain waveform of epileptic patients. Record ‘C' and ‘D' are interictal signals that are recorded using seizure-free intervals. EEG signals in set C are recorded from a region opposite to epileptogenic zone, whereas set D is constructed by recording EEG signals from the epileptogenic zone. On the other hand, set E contains true seizures waveforms.  Figure 2 shows the first 1000 sample points of a randomly chosen EEG waveform from each set.

In this study, we have used all the five sets. Each set indicates one class, and each class consists of 100 instances with each instance having 4097 sampling points. In this research paper, we have studied 2, 3, 4, and 5 class problems. The details of dataset are given in Table 1. In 2-class problem, total instances used are 200 whereas for 3, 4, and 5 classes, 500 instances are considered.

#### 2.1.2. The CHB-MIT Dataset

Another database used to validate the effectiveness of the proposed model is CHB-MIT [21]. It is also an open-source EEG database constructed by Children's Hospital Boston and the Massachusetts Institute of Technology (MIT). It contains EEG noninvasive recordings from 23 pediatric patients, including male patients between the ages of [3, 22] years and female patients with an age range of [1.5, 19] years. These EEG recordings were recorded using the International 10–20 system at a sampling rate of 256 Hz and with 16-bit resolution [19]. The binary classification problem is studied. In total, 1600 instances are considered, 800 for each category. Each instance has a length of 5.0 seconds and contains 1280 sampling points per channel.  Figure 3 shows the first 1000 sampling points of the randomly chosen preictal and ictal, signals from the CHB-MIT database.

### 2.2. Preprocessing

The raw EEG signals obtained from the dataset are contaminated with noise, which can influence the EEG signal's low-frequency spectrum and can cause loss of some useful information. The frequency range of EEG recordings in the Bonn database is 0–86.8 Hz. Frequencies higher than 50 Hz are considered as noise. Therefore, preprocessing of a signal is required to remove the redundant frequency. For this, all the five sets of raw EEG signals obtained from the Bonn dataset are passed through a zero-phase band-pass Butterworth filter of order 2. The Butterworth filter is a signal processing filter, which is used for noise removal. The EEG recordings from both datasets are passed through the Butterworth filter, which filters out slow-frequency components, high frequency noise, and limit the frequency content of the signal to a range of [0.5, 50] Hz.

### 2.3. Discrete Wavelet Transform

EEG time-series signals are nonstationary because of electromagnetic interference between high-frequency oscillators and low-frequency signals generated due to eye blinks and muscle stretching while recording [22]. We can directly use CNN on raw EEG signals to extract features but the noise generated during recording would affect the classification accuracy. Also, the results vary for different datasets. It is quite challenging to capture frequency information during brain activity [23]. From the literature review, we observed that wavelet transform (WT) based methods capture the transient information accurately by providing both time-domain and frequency domain information of a signal [24]. Two of the most commonly used WT methods include CWT and DWT. CWT provides a high level of redundancy, thus, generating a lot of unused information and calculations [25, 26]. DWT addresses the weakness of CWT and provide multiscale representation of EEG signals as shown in Figure 4. The input signal *x*[*n*] is passed through a series of high-pass (HPF) and low-pass filters (LPF) and generates approximate and detailed coefficients at every level. D1, D2, D3, and D4 represent detailed coefficients, whereas A4 is an approximate coefficient.

After the preprocessing step, the Butterworth-filtered signal is fed to the discrete wavelet transform as an input. Discrete wavelet transform decomposes signal into sub-bands. In this paper, we have used the fourth order Daubechies (db4) wavelet as it is the most suitable for epileptic seizure detection and is known for its orthogonality property and its smoothing features [27, 28].

### 2.4. Features Extraction

Previous studies used different feature extraction algorithms to extract features. Some algorithms worked on one dataset, but the features extracted on other dataset classified the instances with lower accuracy. Therefore, instead of manually extracting features, we used the feature extraction part of CNN to extract features. CNNs are the deep neural networks that are specialized to automatically learn the internal representations of the data. They use kernels or filters which are convolved over the entire data to produce feature maps. As mentioned previously we have performed 2-class, 3-class, 4-class, and 5-class classification for the Bonn dataset, and binary classification is performed for the CHB-MIT dataset. One-dimensional CNN is trained using different combinations of kernel numbers and sizes. The parameters on which maximum accuracy is obtained are selected. The learning rate is varied from 0.01 to 0.0001 and the effect is observed. In case of Bonn dataset, we have used only one convolution layer and pooling layer to extract features in a 2-class problem i.e., A vs. E and B vs. E. These features were then flattened to a 1D feature vector, which was then sent to different classifiers for classification. Our main focus is to achieve maximum accuracy with a smaller number of layers.  Figure 5 shows the CNN architecture chosen for the 2-class problem in the Bonn dataset.

For the multiclass problem of the Bonn dataset and the binary classification of CHB-MIT dataset, we have trained 2-layered, 4-layered, and 6-layered CNNs. We observed that the 4-layered CNN architecture performed better in terms of classification accuracy. The general architecture of CNN is the same for all the problems, with a slight variation in the number of kernels used, and is shown in Figure 6.

There are two convolution layers followed by maximum pooling layers. The input layer is convolved with a kernel of convolution layer and generates output known as feature maps. To introduce nonlinearity in the network and faster learning, the ReLU activation function is used. It allows the model to learn faster and overcomes the vanishing gradient problem. After that, a maximum pooling layer is applied to every feature map, which reduces the spatial size of feature maps. Now, CNN has learned the features, but they are in the form of two-dimensional feature maps. After passing through a series of these layers, the feature maps reach the flatten layer, which flattens the feature maps into a one-dimensional feature vector so that they can be fed as an input to the classifiers. For classification, these features are sent to the dense layers of CNN and to ML classifiers. In the classification part of CNN, there are three dense layers. The number of neurons in the first two dense layers is fixed to 50 and 20. The number of neurons in the last dense layer is equal to the number of classes. For example, in a 3-class problem, there are 3 neurons in the last layer.

Table 2 shows the parameters selected for 3, 4, and 5 class problems. Here, *K*, *Ks,* and *S* denotes number of kernels, kernel size and Stride. Similarly, in maximum pooling layer, *Ps* and *S* represent pooling size and stride. The feature maps generated as a result of multiple convolution and pooling layers are converted to a 1-dimensional array which represents the total number of features learnt and is represented by *F*. *N* indicates the number of neurons in each dense layer. The details of how these parameters are adjusted are given in Section 3. The learning rate, epochs and batch-size is set to 0.001, 100, and 12. The *k*-fold cross-validation strategy is employed for CNN training where *k* is set to 10.

### 2.5. Feature Selection

The CNN model learns the features from every training sample. But some of the features are redundant or of less importance. The presence of these irrelevant or redundant features can affect the performance of a network and also increase the data dimensionality [29]. Therefore, we have employed a mutual information (MI) estimator to reduce the curse of dimensionality and processing time by selecting fewer and more relevant features. It is one of the most widely used estimators for feature selection due to its ability to detect nonlinear relationships between the features and the target variable [29]. It measures the amount of information one can obtain from a discrete random variable *A* when a discrete random variable *B* is given. This mutual information is calculated in the following equation:

(1) $$\begin{array}{c} I\left(A;\;B\right)=\underset{b\in B}{\sum }\underset{a\in A}{\sum }p_{\left(A,B\right)}\left(a,b\right)\log\left(\frac{p_{\left(A,B\right)}\left(a,b\right)}{P_{A}\left(a\right)P_{B}\left(b\right)}\right)\text{,} \end{array}$$

where *p*_(*A*, *B*)_ is the joint probability mass function of the discrete random variables *A* and *B*. *p*_*A*_(*a*) an d *p*_*B*_(*b*) represents the marginal probability mass functions of *A* and *B* variables. If the mutual information is 0, then the two variables are strictly independent. The estimator works by computing the MI score of all features with respect to the target variable and selecting the features by comparing their score against some threshold. In this way, MI minimizes the redundancy of the selected features [30]. Different number of features such as 50, 100, 150, 200, and 1000 with maximum information scores have been selected, and their effect is observed on the model's performance.

### 2.6. Classification

The last step is the classification of EEG signals. After feature extraction, feature selection has further reduced the size of data matrix. Now, the features extracted by convolution and pooling layers are passed to fully connected layers. They can also be extracted and sent to other ML classifiers. The brief detail of classifiers used for classification in the following.

  Artificial neural network (ANN) [31, 32] is widely used for processing biomedical signals such as EEG signals [33]. Most of the studies have used ANN for epilepsy detection using EEG signals [34–36]. They are simple neural networks in which each neuron in a hidden layer is connected with all the neurons of the previous layer. We have used a three-layered ANN for feature classification. The first two layers consist of 50 and 20 neurons. In the last layer, the number of neurons is equal to the number of class labels.
  Logistic regression (LR) [37] is another powerful ML algorithm which is used to model dichotomous target variables. The hyperparameters are tuned using “Grid Search CV” library of Python.
  Random forest (RF) [35] is an ensemble-based ML algorithm which uses a multitude of decision trees in which each tree behaves as a classifier and a certain weight is given to the output of all trees. We have chosen 100 decision trees using 10-fold cross-validation. They predict a particular class based on the input features. After prediction, a consensus is carried out among all the outputs to predict a class label.
  Support vector machine (SVM) [38] uses a kernel trick which takes a low dimensional input space and transforms it into a higher dimensional space and then classifies this data using a linear decision boundary. In our study, we have used radial basis function (RBF) kernel. The classifier is trained on the training examples and outputs an optimal hyperplane which is able to classify new unseen examples. In our study, the regularization parameter (*C*) is set to 100 and gamma value is set to 0.0001.
  Gradient boosting classifier (GB) [39] is also an ensemble technique that is based on the assumption that many weak learners, when combined generate a stronger learning model. Rather than fitting a predictor to the data at each iteration, it fits a new predictor to the residual errors of the previous prediction. We have used 400 estimators, and the learning rate is set to 0.001.
  k-nearest neighbors (k-NN) [40, 41] is a nonparametric supervised algorithm. It saves all training data and then makes future predictions based on the similarities between each input sample and each training example. The algorithm takes a fixed positive integer *k* as an input. It then classifies a new data point *x*_0_ by first defining the *k* points in the training set that are closest to this new data point and then computes the minimum distance between the neighboring *k* points and *x*_0_ for very class label [19]. The most frequent label among the labels of *k* points will be assigned to *x*_0_. In this case, we have used *k* = 3 and Manhattan distance as a distance metric.
  Stochastic gradient descent (SGD) [42] implements stochastic gradient descent (SGD) learning to train a linear model. In machine learning, the learning process produces the function by processing the training set's samples. This function maps input values to one of the classes. SGD is an optimization technique that seeks to discover the coefficient of this function under a condition that minimizes the cost margin. The hyperparameters of SGD are chosen using GridsearchCV and 10-fold cross-validation. After training data on different combinations of parameters, the parameter selected by GridsearchCV are given in Table 3.
  Stacking ensemble classifier [43] is an ensemble learning technique that builds a new model using predictions from multiple weak classifiers known as base learners or base models. These weak classifiers are trained in parallel, and their predictions are used to train a meta learner that predicts the final output class. In our study, we have used SVM and k-NN classifiers as base learners and logistic regression as a meta learner. Tenfold cross-validation is employed for model training.

### 2.7. Evaluation Metrics

Following evaluation metrics are calculated to evaluate the performance of model. Accuracy is a ratio of correctly predicted labels to the total predicted labels and is given by the following equation:

(2) $$\begin{array}{c} Accuracy=\frac{\left(TP+TN\right)}{TP+FP+FN+TN}\text{,} \end{array}$$

where TP represents true positives and are correctly predicted positive labels, TN represents true negatives and are correctly identified negative examples. On the other hand, FP and FN represents false positives or misclassified positive labels and false negatives or misclassified negative labels, respectively.

Precision is the ratio of true positives (TP) to the sum of true positives (TP) and true negatives (TN). It indicates how confident our model is when it classifies a label as positive. Mathematically,

(3) $$\begin{array}{c} Precision=\frac{TP}{TP+FP}\text{.} \end{array}$$

Precision measures how many predicted positive examples are actually positive. Higher the precision, more confident is our model.

Recall is another evaluation metric used to identify how correctly or model has identified actual positive labels. Recall is the ratio of correctly predicted positive classes to all observations in actual class and is given by the following equation:

(4) $$\begin{array}{c} Recall=\frac{TP}{TP+FP}\text{.} \end{array}$$

Higher the recall, more accurate will be our model.

*F*1-score is defined as the weighted average of both recall and precision. It is calculated by using the following equation:

(5) $$\begin{array}{c} F1\;Score=\frac{2\times \left(Precision\times Recall\right)}{\left(Precision+Recall\right)}\text{,} \end{array}$$

*F*1-score with value near to 1 indicates that the model has low false positives and false negatives. *F*1-score with 0 value represents worst model.

## 3. Experiments and Results

The performance of the proposed model is assessed on the Bonn University and CHB-MIT dataset.

### 3.1. Hyperparameter Tuning of CNN Architecture

In this study, we have used the feature extractor part of CNN for extracting features. The architecture of CNN is selected by varying the number of layers, number of kernels, kernel sizes, and so on. With a 2-layered architecture in the binary classification problem for Bonn dataset, we obtained more than 95% accuracy. But, for multiclass problems, we obtained below 90% accuracy by using only 2-layers. Therefore, we tried 4-layered and 6-layered architecture. The results were almost the same for both architectures, but the 6-layered architecture required more layers which in turn increases the number of parameters. Similarly, hyperparameters are adjusted by observing their effect on classification accuracy. Different activation functions are tried in all layers, and the learning rate is varied. Then the effect of increasing the numbers of kernels in all layers is studied.  Figure 7 shows the effect of different number of kernels in the convolution layers on the classification accuracy. The SGD optimizer is used with a learning rate of 0.001. For a binary problem, binary cross-entropy is used for measuring training loss and categorical cross-entropy for a multiclass problem.

After selecting the number of kernels, we changed the kernel size in all layers and observed the effect on accuracy. The results obtained are shown in Figure 8. The *x*-axis represents the number of kernels in layer 2 and *y*-axis represents the number of kernels in layer 1, whereas *z*-axis represents the accuracy obtained. The last dense layer uses softmax activation function which predicts the probabilities of all classes.

In the above figure, the *x*-axis or layer 1 represents the size of kernels in convolution layer 1, whereas *y*-axis or layer 2 indicates the size of kernels in convolution layer 2. The pooling size and stride in maximum pooling layer is set to 2. When it is changed to 4, the accuracy almost remained same but the number of features learnt by CNN is reduced. This, in turn, reduces the time needed to classify these features and number of parameters in dense layer. The adjusted parameters are given in Table 2.

### 3.2. Experimental Results

First of all, 2-class problem is studied. In case of Bonn dataset, a total of 500 EEG instances with 4097 sampling points are considered. Typical EEG waveforms of the considered classes are shown in Figure 5. The EEG waveforms are first preprocessed using the Butterworth filter of order 2 in a range of 0.5–50 Hz. The same process is repeated with the EEG signals obtained from the CHB-MIT database. DWT is a widely used feature extractor for the analysis of time-series data as confirmed by different studies in the literature. It makes the hidden features of data more apparent. Therefore, we applied DWT to the Butterworth-filtered signals. The preprocessed signals were then decomposed into approximate and detailed coefficients using Daubechies (db4) discrete wavelet transform. In the relevant literature, different feature extraction algorithms have been used to extract features from these coefficients. But, we have replaced the manual feature extraction process by CNN. CNN process this data and extract features which were then flattened to pass them dense layers for epileptic seizures classification. Instead of passing these feature maps to the dense layer, we extracted them and passed them directly to the machine learning classifiers for classification. The 10-fold cross-validation is employed in this study for accurate tunning of hyperparameters.  Table 4 shows the results obtained by directly passing the feature maps to ML classifiers.

It can be seen from the above table the proposed architecture classified 2-classes of Bonn dataset with 99.5 and 99% accuracies. As the number of classes increases, the accuracy decreases but remains comparable to the accuracy achieved in previous studies.

Some features are of less importance or are redundant. In mobile healthcare applications, these features are sent to the cloud or a server for further processing. The greater the number of features, the more power and bandwidth will be consumed. The increase in the number of features also increases the training time and increases the risk of model overfitting. Therefore, the redundant features should be discarded to increase the processing speed of classifiers, reduce memory storage, and power consumption. We studied the effect of number of features on the performance of the model. Different numbers of features are selected using the mutual information (MI) score and fed to machine learning classifiers and their accuracies are reported. Mutual information gain selects *k* best features based on the information gain score. In case of A and E classification, all ML classifiers have 100% predicting accuracy. The results for other combinations are shown in Figures 9(a)–9(f).

It can be seen from the graph that even at 50 features, the model achieved 100% accuracy on 2-class problem for Bonn dataset and 97.2% for CHB-MIT data.  Table 5 shows the maximum accuracy reported along with minimum number of features and other evaluation metrics for multiclass problems. k-NN predicted the three classes i.e., normal, interictal and ictal with 97.8% accuracy. But when bagging k-NN is used, the accuracy increased to 99%. Bagging k-NN fit k-NN to random subsets of the original dataset and then aggregate their individual predictions (either by voting or average) to generate a final prediction.

## 4. Discussion

From the results provided in the previous section, it can be seen that the proposed solution efficiently detected five classes.  Table 6 illustrates the comparison of previous studies with the proposed approach. Many previous works have been carried out to detect epileptic seizures with time-series signals such as EEG signals.

EEG signals have the ability to measure the electrical activity of the brain efficiently, but they have poor spatial resolution and often get contaminated with noise and artefacts during signal acquisition. The approach proposed in [1] used the Chebyshev IIR filter for preprocessing. The study conducted in [6] used empirical mode decomposition (EMD) and intrinsic mode function (IMF) for preprocessing. The solution presented in this paper used the Butterworth filter to remove noise from the signals. Later, discrete wavelet transform is applied to obtain a time-frequency representation of an EEG signal. The training of traditional machine learning-based approaches requires feature extraction, for which various methods have been proposed in the literature [1, 6, 7, 9, 10]. These handcrafted features require the expert knowledge of the data and take time to choose the best features for good classification performance.

As compared to the previous studies [1, 9, 10, 14], which extracted features using wavelet analysis of EEG waveforms, the proposed approach uses CNN for feature learning. Studies conducted in [3, 12–14] used CNN to automatically learn the feature by passing the training data through multiple convolutions and subsampling operations. However, the feature extraction using CNN is a time taking process and requires a large number of training samples for appropriate tunning of hyperparameters. Similarly, recurrent neural networks (RNN) and long short-term memory (LSTM) networks have been used in the literature for the analysis of time-series signals. RNN have a gradient vanishing problem and are unable to learn long-term dependencies. LSTM overcomes the shortcomings of the RNN network and is used in the literature for epileptic seizures classification [17, 18]. Hu et al. [18] extracted statistical features using local mean decomposition and trained a Bi-LSTM on these features. Their model achieved 93% sensitivity on the CHB-MIT dataset, whereas we have 97% sensitivity. More training samples can also lead to overfitting of the model.

Many machine learning algorithms have been found to have good generalization ability and can even solve the problems having small training samples [47]. Moreover, the performance of the CNN classifier can be greatly enhanced by the appropriate selection of hyperparameters such as number of filters, filter size, kernel size, pooling size, learning rate, epochs, activation function, optimizer, and batch size. Although the setting of these parameters is difficult, our approach uses CNN combined with different machine learning classifiers to detect epileptic seizures and has improved the classification accuracy along with the generalization ability of the classifier. The binary classification problem involves classification of A and B sets from the E set. Our model is able to achieve 100% accuracy on the binary classification problem.

Jiang et al. proposed a feature extraction technique using symplectic geometry decomposition with 100% and 99% accuracy on the 2-class problem of both datasets and 99% accuracy on the 3-class problem. But they have not tried 4-class and 5-class problem. For multiclass problem, we achieved state-of-the-art accuracy. The presented model achieved an accuracy of up to 99.33% on 3-class problem, which is obviously better than the models in [3, 4], which are based on CNN only. On the other hand, 5-class problem is more complicated as compared to 2-class and 3-class problems. Deep learning-based architectures proposed in the literature extracts large number of features for classification. As discussed previously, these features require more memory, time, and bandwidth for the processing of highly dimensional data matrix. Some of the features are redundant or irrelevant or noisy and can negatively impact the performance of a network. Therefore, appropriate feature selection is essential. One of the widely used feature selection estimators used in machine learning applications is mutual information gain (MI) [48]. The model selected different number of features from 50 to 1000 using MI estimator and observed their effect on the accuracy. The proposed model achieved an accuracy of 94% and 93% on 4- and 5-class problem. This accuracy is very close to the results of the 5-class problem in [3] and [13].

## 5. Conclusions

The CNN-based model is presented in this paper, which along with the combination of different machine learning algorithms predicts epileptic seizures. The EEG waveforms are filtered using the Butterworth filter and passed to CNN for feature learning. The transfer learning approach is used in which the dense layers are replaced by the machine learning classifiers such as support vector machine (SVM), random forest (RF), gradient boosting classifier (GB), logistic regression (LR), and so on. In addition, it uses MI-based feature selection estimator which selects only relevant features and passes them to the classification model. Feature selection helps to avoid the curse of dimensionality. In contrast to the conventional equivalents, it replaces the manual feature extraction process and improves the generalization ability of the classifier. The proposed approach achieved highest accuracy of 100% and 97% on 2-class problem of the Bonn dataset and the CHB-MIT dataset, whereas for the 3-class problem, bagged k-NN performed very well with 99% accuracy. SVM and ensemble classifiers predicted 4- and 5-classes with 94.4% and 93.6% accuracies, respectively. The solution presented in this paper is able to achieve accuracy close to the accuracy reported in previous studies.

In future studies, other potential EEG datasets will be considered for confirming the robustness of the proposed methodology. Additionally, the feasibility of incorporating the other decomposition techniques, like empirical mode decomposition and tunable Q-factor wavelet transform, in the suggested method will also be investigated.

## Figures and Tables

**Figure 1:** Block diagram.

**Figure 2:** Typical EEG waveforms in Bonn dataset.

**Figure 3:** Typical EEG waveforms in CHB-MIT dataset.

**Figure 4:** Decomposition of EEG signal into sub-bands using db4 wavelet.

**Figure 5:** CNN architecture for 2-class problem of Bonn dataset.

**Figure 6:** CNN architecture for multiclass problem and binary classification for Bonn and CHB-MIT dataset.

**Figure 7:** Effect of number of kernels on the classification accuracy for (a) 3-class, (b) 4-class, and (c) 5-class problem of Bonn dataset and (d) 2-class of CHB-MIT dataset.

**Figure 8:** Effect of kernel size on the classification accuracy for (a) 3-class, (b) 4-class, and (c) 5-class problem.

**Figure 9:** Effect of features reduction on the accuracy of ML classifiers for (a) A–E set, (b) B–E set, (c) AB–CD–E, (d) AB–C–D–E, (e) A–B–C–D–E, and (f) CHB-MIT.

**Table 1:** Construction of dataset based on the classification problem.

Classification problems	Sets combination
2-Class	A vs. E
	B vs. E

3-Class	AB vs. CD vs. E
4-Class	AB vs. C vs. 9D vs. E
5-Class	A vs. B vs. C vs. D vs. E

**Table 2:** CNN hyperparameters for 3, 4, and 5-classes problems.

Bonn datasets					CHB-MIT datasets
Layers	2-class	3-class	4-class	5-class	2-class
Conv.	*K* = 4, *Ks* = 3, *S* = 1	*K* = 10, *Ks* = 4, *S* = 1	*K* = 11, *Ks* = 5, *S* = 1	*K* = 11, *Ks* = 5, *S* = 1	*K* = 11, *Ks* = 3, *S* = 1
Max. Pooling	*Ps* = 4, *S* = 4	*Ps* = 4, *S* = 4	*Ps* = 4, *S* = 4	*Ps* = 4, *S* = 4	*Ps* = 4, *S* = 4
Conv.	—	*K* = 5, *Ks* = 5, *S* = 1	*K* = 9, *Ks* = 5, *S* = 1	*K* = 7, *Ks* = 5, *S* = 1	*K* = 7, *Ks* = 11, *S* = 1
Max. Pooling	—	*Ps* = 4, *S* = 4	*Ps* = 4, *S* = 4	*Ps* = 4, *S* = 4	*Ps* = 4, *S* = 4
Flatten	*F* = 7720	*F* = 2405	*F* = 4329	*F* = 3367	*F* = 1043
Dense	*N* = 50	*N* = 50	*N* = 50	*N* = 50	*N* = 50
Dense	*N* = 20	*N* = 20	*N* = 20	*N* = 20	*N* = 20
Dense	*N* = 2	*N* = 3	*N* = 4	*N* = 5	*N* = 2

**Table 3:** SGD hyperparameters.

Parameters	Bonn datasets	CHB-MIT datasets
Alpha	0.001	0.01
Eta0	100	1
Learning rate	Optimal	Adaptive
Loss function	Modified_huber	Hinge
Penalty	Elastic net	Elastic net

**Table 4:** Summary of results obtained using different machine learning classifiers.

Datasets	No. of classes	Classes names	ANN	LR	RF	SVM	GB	k-NN	SGD	Ensembles
Bonn dataset	2	A–E	97.5	99.5	99.5	96.5	97	92	99.5	97
		B–E	97	99	99	95	95	91.5	99	96
	3	AB–CD–E	98	97.4	95	97.8	97.4	98.2	97.6	97.8
	4	AB–C–D–E	89.6	94.6	92	93.2	93.8	93.2	94.4	92.8
	5	A–B–C–D–E	87	92.4	89.4	93.2	88.8	89	89	92.2

CHB-MIT dataset	2	Ictal–Preictal	94.4	91.7	92.4	95.7	94.6	96.8	87	97

**Table 5:** Evaluation metrics result obtained on prediction of multiclass problems.

Classes	Number of features	Classifier	Accuracy (%)	Precision	Recall	*F*1-score
A–E	50	RF	100	1.0	1.0	1.0
B–E	100	RF	100	1.0	1.0	1.0
AB–CD–E	700	Bagged k-NN	99	0.99	0.99	0.99
AB–C–D–E	1000	LR	94.4	0.95	0.94	0.94
A–B–C–D–E	3367	SVM	93.6	0.94	0.94	0.94
Ictal vs. Preictal	500	Ensemble	97.1	0.97	0.97	0.97

**Table 6:** Comparison of previous studies conducted for epilepsy detection.

Study	Features extraction	Classification method	Datasets	Classes	Accuracy (%)
[1]	Chebyshev IIR filter, discrete wavelet transform	SVM	Bonn	2	96
		ANN			98
[3]	None	CNN	Bonn	2	99.52
				3	96.97
				5	93.55
[4]	None	CNN	Bonn	3	88.67
[6]	Empirical mode decomposition (EMD), intrinsic mode function (IMF)	Classification and regression tree (CART)	Bonn	3	93.55
[7]	Recurrence quantification analysis (RQA)	SVM	Bonn	3	95.60
[8]	Channel selection and statistical feature extraction	Ensemble	CHB-MIT	2	89.02%
[9]	Tunable-Q wavelet transform (TQWT)	Random Forest (RF)	Bonn	3	99
[10]	Multiscale PCA, wavelet packet decomposition	SVM	Bonn	3	99.70
[11]	Discrete wavelet transform, temporal and spectral features	Fuzzy rough	CHB-MIT	2	92.79%
		Nearest neighbor			
[12]	None	1D-pyramidal CNN	Bonn	3	99.1
[13]	None	1D-feature fusion CNN	Bonn	3	98.67
[14]	CWT	CNN	Bonn	2	100
				3	99
				4	91.50
				5	93.60
[44]	Time-frequency analysis (TFA)	ANN	Bonn	2	100
				5	89
[45]	Symplectic geometry eigenvalues	SVM	CHB-MIT	2	99.62
[46]	Adaptive-rate FIR filtering and DWT + MI-based feature selection	Ensemble of MLP, k-NN, SVM, BG, and RF	Bonn	2	100
		—		3	99.50
				4	96
				5	92
			CHB-MIT	2	99.38
Our approach	CNN	ML classifiers	Bonn	2	100
				3	99.33
				4	96
				5	94
	—	—	CHB-MIT	2	97.1

## Data Availability

The datasets used in this paper are publicly available via the following links: (http://epileptologie-bonn.de/cms/upload/workgroup/lehnertz/eegdata.html) and (https://physionet.org/physiobank/database/chbmit/).
